# TXI: Texture and Color Enhancement Imaging for Endoscopic Image Enhancement

**DOI:** 10.1155/2021/5518948

**Published:** 2021-04-07

**Authors:** Tomoya Sato

**Affiliations:** Department of Advanced Imaging System Technology, Olympus Medical Systems Corporation, 2951 Ishikawa-machi, Hachioji-shi, Tokyo 192-8507, Japan

## Abstract

Recognition of lesions with subtle morphological and/or color changes during white light imaging (WLI) endoscopy remains a challenge. Often the endoscopic image suffers from nonuniform illumination across the image due to curvature in the lumen and the direction of the illumination light of the endoscope. We propose an image enhancement technology to resolve the drawbacks above called texture and color enhancement imaging (TXI). TXI is designed to enhance three image factors in WLI (texture, brightness, and color) in order to clearly define subtle tissue differences. In our proposed method, retinex-based enhancement is employed in the chain of endoscopic image processing. Retinex-based enhancement is combined with color enhancement to greatly accentuate color tone differences of mucosal surfaces. We apply TXI to animal endoscopic images and evaluate the performance of TXI compared with conventional endoscopic enhancement technologies, conventionally used techniques for real-world image processing, and newly proposed techniques for surgical endoscopic image augmentation. Our experimental results show that TXI can enhance brightness selectively in dark areas of an endoscopic image and can enhance subtle tissue differences such as slight morphological or color changes while simultaneously preventing over-enhancement. These experimental results demonstrate the potential of the proposed TXI algorithm as a future clinical tool for detecting gastrointestinal lesions having difficult-to-recognize tissue differences.

## 1. Introduction

Endoscopic screening plays a significant role in early lesion detection for reducing gastrointestinal cancer-related mortality. Colorectal cancer is the most common gastrointestinal cancer worldwide, and over 1.8 million new cases and 862,000 deaths were reported in 2018 [1]. In colorectal cancer, early detection of colorectal polyps during total colonoscopy is important to avoid interval cancer, and the improvement of the adenoma detection rate by 1% is associated with a 3% decrease in the rate of the interval cancer [2]. Gastric cancer is the second most common gastrointestinal cancer worldwide and early detection is useful for improving the 5-year disease-specific survival rate [3]. The current standard practice for colorectal polyp detection and gastric cancer detection is endoscopy using white light imaging (WLI); however the performance of WLI for detecting early colorectal and gastric lesions is not satisfactory [4, 5]. For example, colonoscopy studies suggest the miss rate for colorectal polyps may be as high as 22% to 26% [5]. Polyps having slight morphological change such as flat or depressed polyps and polyps that are pale in appearance or have subtle color changes are likely to be overlooked [6–8].

To improve detection performance, several clinical investigations regarding the usefulness of image-enhanced endoscopy (IEE) [9] have been conducted. Optical image-enhanced technology such as narrow band imaging (NBI) [10] has been extensively studied. In the stomach, the benefit of NBI for early gastric cancer detection is uncertain as a recent multicenter randomized controlled trial did not find an increase in detection rate with the use of NBI over WLI [11]. In the colon, NBI may assist an endoscopist to achieve a higher adenoma detection rate over WLI but only when bowel preparation is optimal [12]. Accordingly, there has been growing interest in developing new technology for improving the detection performance.

In this paper, we investigate an endoscopic image enhancement technology designed with the intent to improve detection of gastrointestinal lesions. As mentioned above, it is difficult to recognize lesions with subtle morphological and/or color changes in WLI. The endoscopic image often suffers from nonuniform illumination due to curvature in the lumen and the direction of the illumination light of the endoscope. The nonuniform illumination can make observation difficult because distant area may appear darker. We propose a new image enhancement technology to resolve these drawbacks called texture and color enhancement imaging (TXI). TXI is designed to enhance three image factors in WLI (texture, brightness, and color) to define subtle tissue differences clearly.

Several image processing techniques have been proposed for resolving nonuniform illumination in real-world images. Histogram equalization (HE) and gamma correction (GC) are well-known and widely used techniques because of their simple algorithms. In HE, the histogram of the entire image is adjusted to balance the grayscale values and GC enhances the brightness and contrast by expanding the dark regions and compressing bright regions. However, the main drawback of these methods is that each pixel in the image is treated individually without considering neighboring pixels resulting in an output image inconsistent with the input image. To resolve the above problems, adaptive image enhancement techniques that treat each pixel relative to their surroundings have been proposed. For example, the retinex theory [13] which is based on human visual characteristics has been widely applied in real-world image processing to enhance low-light brightness. In the retinex theory, the original image is split into two layers, a base layer and a detail layer, and each layer is processed to improve nonuniform illumination. Wang et al. [14] proposed a colored image correction method based on nonlinear functional transformation according to the multiscale retinex model. Okuhata et al. [15] proposed an estimation of the base layer by using the variational retinex model and applying GC to the base layer of endoscopic images. Luo et al. [16] demonstrated the use of a modified multiscale retinex model on surgical endoscopic images in which only the detail layer was used for resolving the nonuniform illumination. However, in these methods, it is difficult to maintain the brightness and color fidelity of the image as well as HE or GC alone. For example, the image brightness in blight regions is compressed by applying GC to the base layer in [15], and the base layer which includes information of image brightness and color is completely excluded in [16]. In gastrointestinal endoscopy, WLI is used as the standard baseline for observation, so it is crucial to maintain consistency of the brightness and color in the original WLI image for the comfort and familiarity of the physician.

In order to resolve the above drawbacks, we propose an image processing technology modifying retinex-based processing to enhance subtle tissue differences with maintenance of WLI appearance. Moreover, we also propose combination of the retinex-based enhancement with color enhancement for greatly enhancing color tone to aid in easier recognition of subtle color differences. The novelty of this work is to improve not only the illumination nonuniformity in the image, which was proposed in related works [14–16], but also enhance subtle tissue differences by applying retinex-based algorithms and color enhancement algorithm to gastrointestinal images while maintaining image naturalness (WLI appearance).

In this paper, we present the TXI algorithm and quantitative assessment metrics of endoscopic images for validating TXI performance. Additionally, we apply TXI to animal endoscopic images and evaluate the performance of TXI by compared against conventional IEE methods used in clinical practice such as structure enhancement [9] and index of hemoglobin (IHb) color enhancement [9], real-world image processing techniques such as HE, and a newly proposed technique [16] for surgical endoscopic image augmentation. The results from these animal experiments show that TXI provides a balance of improving image features important for the physician searching for abnormalities (selective increase in brightness, greater color separation, and texture enhancement) while minimizing gross changes that may negatively impact familiarity (naturalness).

## 2. Approach

This section presents the TXI algorithm and definitions of quantitative assessment metrics for endoscopic image evaluation. In TXI, after estimating the base and the detail layers, a partial brightness adjustment is applied to the base layer with maintenance of the brightness in bright areas and color balance of RGB components. Since the slight morphological and color changes are included in the detail layer, the contrast enhancement of such changes is achieved by using the detail layer. For detail enhancement, we propose an important modification in the application of the retinex-based method to endoscopic images. In endoscopic images, several bright spots are often present due to specular reflection. Since bright spots are generally very small regions and significantly high contrast, these are not extracted in the base layer but in the detail layer corresponding to local contrast of brightness and color in the scene. Thus, enhancement of the detail layer induces strong augmentation of the bright spots, and such enhanced spots may obscure the image and lead to missed lesions. To resolve this drawback, we propose a method to remove the bright spots from the detail layer by including the spots in the base layer.

### 2.1. TXI Algorithm

TXI is designed to enhance three image factors (texture, brightness, and color) by applying the retinex theory. The basis of this theory is to decompose an image into two distinct layers according to human visual characteristics: a base layer which represents the illumination component in the scene and a detail layer corresponding to local contrast of brightness and color in the scene. The local contrast of the sensor can be decreased by tone-mapping since the larger dynamic range of the sensor is mapped into a smaller range. The aim of this theory is to prevent such contrast reduction by compression of the base layer while maintaining the detail layer.

The flowchart of TXI is shown in Figure 1. TXI consists of the following six processes. The input image is split into the base layer and the detail layer in Step 1 by using a single-scale retinex algorithm (SSR) [17]. In Step 2, the brightness in dark regions of the base layer is corrected. It is difficult to adjust the brightness selectively in dark regions of the image by light source control because it is applied across the entire image and can lead to halation in brighter areas. On the other hand, since the base layer corresponds to the illumination component, the partial brightness control in the image can be achieved through processing techniques. Texture and color are enhanced in Steps 3–5. The dynamic range of the base layer alone is compressed in Step 3 to maintain the local contrast, important for slight morphological or color changes included in the detail layer. In Step 4, texture enhancement is applied to the detail layer for enhancing subtle contrast. The compressed base layer and the enhanced detail layer are recombined in Step 5 to produce a TXI image for immediate display as TXI mode2 or for further processing. The output image from Step 5 has its color tone enhanced in the final Step 6. The color enhancement algorithm is designed to expand color difference in the image particularly between red and white hues. The output from Step 6 is the TXI mode1. There are two settings for TXI: mode1 with color enhancement and mode2 without color enhancement, which has an appearance closer to WLI color tone.

**Step 1 .**

Split into two layers

SSR [17] and multiscale retinex algorithm (MSR) [18] are well-known as simple retinex-based algorithms. In this work, we use SSR because of its simplicity and easy implementation.

SSR is given by

(1) $$\begin{array}{c} \log D_{c}\left(x,y\right)=\;\log I_{c}\left(x,y\right)-\log B_{c}\left(x,y\right), \end{array}$$

where (*x*, *y*) is a pixel on input image **I**_*c*_ with three color channels of red, green, and blue (*c* ∈{*R*,  *G*,  *B*}). **D**_*c*_ and **B**_*c*_ represent the detail layer and the base layer, respectively. According to SSR, the base layer can be calculated by convolving Gaussian filter with **I**_*c*_. However, there is a drawback of applying SSR using Gaussian filter, which is a halo artifact occurring around edges in the image. The methods for calculating the base layer using an edge-preserving filter to resolve this drawback were reported in [19, 20]. In this work, we use an edge-preserving filter instead of a Gaussian filter, and the base layer is derived using

(2) $$\begin{array}{c} B_{c}\left(x,y\right)=\frac{1}{k_{p}}\sum_{q\in \Omega }f\left(\left\|p-q\right\|\right)g\left(\left\|I_{c}\left(x,y\right)-I_{c}\left(u,v\right)\right\|\right)I_{c}\left(u,v\right), \end{array}$$

where **p** and **q** are pixel locations, and **p** = (*x*, *y*) and **q** = (*u*, *v*). *k*_*p*_ is a normalization term:

(3) $$\begin{array}{c} k_{p}=\sum_{q\in \Omega }f\left(\left\|p-q\right\|\right)g\left(\left\|I_{c}\left(x,y\right)-I_{c}\left(u,v\right)\right\|\right), \end{array}$$

where *f* is a Gaussian function in the spatial domain and *g* is a Gaussian for intensity domain.

As mentioned above, bright spots generally can occur in the endoscopic images. Since the bright spots are very small regions and high contrast, these are not extracted in the base layer by (2) but in the detail layer. It is necessary to remove these spots from the detail layer to avoid over-enhancement of the spots. This is conducted by using

(4) $$\begin{array}{c} B_{c}\left(x,y\right)=\left(1-w\right)B_{c}\left(x,y\right)+wI_{c}\left(x,y\right), \end{array}$$

(5) $$\begin{array}{c} \begin{array}{c} w=1\;\left(\left(x,\;y\right)\in \Omega \right),\;\\ w=0\;\left(\left(x,\;y\right)\notin \Omega \right), \end{array} \end{array}$$

where Ω is the area of the bright spots. The bright spots in the image can be included in the base layer by using (4). By using (1) and (4), the detail layer is derived again using

(6) $$\begin{array}{c} \log D_{c}\left(x,y\right)=\left\{\begin{array}{cc} 0, & \left(\left(x,y\right)\in \Omega \right),\\ \log I_{c}\left(x,y\right)-\log B_{c}\left(x,y\right)\;, & \left(\left(x,y\right)\notin \Omega \right). \end{array}\right) \end{array}$$

Thus, **D**_*c*_=1 within the bright spots.

**Step 2 .**

Brightness adjustment

The correction of brightness in dark area is conducted by using

(7) $$\begin{array}{c} B_{\max}^{\prime }\left(x,y\right)=\left\{\begin{array}{cc} \frac{h}{h^{\alpha }}B_{\max}^{\alpha }\left(x,y\right)\;, & \left(B_{\max}<h\right),\\ B_{\max}\left(x,y\right), & \left(B_{\max}\geq h\right), \end{array}\right) \end{array}$$

where *h* is a threshold parameter, *α* is a brightness correction parameter, and **B**_max_ is the maximum intensity of the base layer in *R*, *G*, and *B* value of each pixel. A higher *h* value represents higher brightness level of the correction target, and a smaller *α* indicates stronger gain in the dark region. These values are empirically determined. At first, we tested *α* = 1/2 and *h* from 1/5 max (*Ic*) to 3/4 max (*Ic*) to find suitable *h* value. We found that *h* = 1/4 max (*Ic*) shows good performance balancing of visualization in dark area and bright area. Then, we tested *α* from 1 to 1/2 and found that *α* = 1/1.4 shows relatively good performance balancing image noise and visualization in dark area. Here, max (**I**_*c*_) represents maximum intensity value among *R*, *G*, and *B* channels. In (7), the base layer with smaller intensity than *h* is corrected according to *α* for increasing brightness in dark areas only. The corrected base layer **B ***'*_*c*_ is derived using

(8) $$\begin{array}{c} B_{c}^{\prime }\left(x,y\right)=M\left(x,y\right)B_{c}\left(x,y\right), \end{array}$$

where **M** (*x*, *y*) is a gain map which represents gain value for the correction in each pixel:

(9) $$\begin{array}{c} M\left(x,y\right)=\frac{B_{\max}^{\prime }\left(x,y\right)}{B_{\max}\left(x,y\right)}. \end{array}$$

In (8), each color channel of the base layer is multiplied by the same gain value. Thus, the color balance which is the ratio in each color channel can be retained, and the brightness correction can be performed while maintaining the color tone of the input image.

**Step 3 .**

Tone-mapping

Tone-mapping is applied to the corrected base layer by using the same function currently used in the chain of endoscopic image processing. Since tone-mapping is generally a nonlinear process, it requires the same tone-mapping function for guaranteeing color reproduction. The base layer after tone-mapping **B**_*c*_^″^is expressed as

(10) $$\begin{array}{c} {B^{\prime \prime }}_{c}\left(x,y\right)=\gamma \left({B^{\prime }}_{c}\left(x,y\right)\right), \end{array}$$

where *γ* is the tone-mapping function currently used in the tone-mapping in the chain of the endoscopic image processing. *γ* is a function similar to the general tone curve function used in gamma correction (GC).

**Step 4 .**

Texture enhancement

Texture enhancement is conducted by using

(11) $$\begin{array}{c} {D^{\prime }}_{c}\left(x,y\right)=D_{c}{\left(x,y\right)}^{g}, \end{array}$$

where **D**′_*c*_ is the enhanced detail layer and *g* is an enhancement parameter. While larger *g* values make it possible to enhance the local contrast, setting it too high may cause over-enhancement. Enhancement parameter *g* is empirically determined. We tested *g* from 1.0 to 2.0 to find suitable *g* value. We found that *g* = 1.2 shows relatively good performance of visualization of the local contrast while suppressing over-enhancement. As shown in (1), the detail layer represents the local contrast which is the difference between the input image and the base layer. Thus, **D**_*c*_(*x*, *y*) = 1 when **I**_*c*_(*x*, *y*) =  **B**_*c*_(*x*, *y*) where no local contrast exists. On the other hand, **D**_*c*_(*x*, *y*) has greater or less value based on 1 when **I**_*c*_(*x*, *y*) ≠ **B**_*c*_(*x*, *y*) where there is local contrast. Therefore, the local contrast resulting from morphological or color changes can be enhanced by (11). Moreover, within the bright spots, **D**_*c*_(*x*, *y*) = 1 by (6), thus, these spots are not influenced by (11), which can prevent over-enhancement of these spots.

**Step 5 .**

Image stacking

The base layer after tone-mapping and the enhanced detail layer are recombined using

(12) $$\begin{array}{c} \log O2_{c}\left(x,y\right)=\log B_{c}^{\prime \prime }\left(x,y\right)+\log D_{c}^{\prime }\left(x,y\right), \end{array}$$

where **O**2_*c*_ is TXI mode 2 output.

**Step 6 .**

Color enhancement

Color enhancement is then applied to the TXI mode2 output for more clearly defining slight color contrast. In particular, pale or red areas are enhanced which is important information for early lesion detection. The color difference Δ*E* is used as a metric of the color contrast in gastrointestinal endoscopic image [21]. Δ*E* is defined as the Euclidean distance between two arbitrary points in CIE 1976 La*∗*b*∗* space, which corresponds to color change perceived by the human visual system. Thus, color enhancement is designed to expand Δ*E* especially between red and white color by directly enhancing color tone in CIE 1976 La*∗*b*∗* space. Color enhancement is conducted in the following manner:

- RGB output of TXI mode2 is converted to CIE1976 La*∗*b*∗*
- The tone in *a∗* is expanded by *C* (*s*) for enhancing color contrast especially between red and white color
- The output from (b) is converted back to RGB output

Let us define *a∗* image and extended *a∗* image as **A** and **A**′, and **A**′ is derived using

(13) $$\begin{array}{c} A^{\prime }\left(x,y\right)=C\left(A\left(x,y\right)\right), \end{array}$$

(14) $$\begin{array}{c} C\left(s\right)=\left\{\begin{array}{c} a_{n}s+b_{n}\;\left(0\leq s<s_{2}\right)\;\left(n=0,1\right),\\ s\;\left(s<0,\;s\geq s_{2}\right), \end{array}\right) \end{array}$$

(15) $$\begin{array}{c} a_{n}=\frac{\left(t_{n+1}-t_{n}\right)}{\left(s_{n+1}-s_{n}\right)}\;,\;\left(n=0,\;1\right), \end{array}$$

(16) $$\begin{array}{c} b_{n}=t_{n+1}-a_{n}s_{n+1},\;\left(n=0,\;1\right). \end{array}$$

As shown in (14), *C* (*s*) is defined as a linear function composed of some polygonal lines due to its easy implementation. The tone in *a∗* is expanded by using *C* (*s*), and a range between *s*_1_ and *s*_*2*_ represents expansion target range. Coordinates of [*s*_*n*_, *t*_*n*_] are empirically determined. While a larger target range between *s*_*1*_ and *s*_*2*_ and a larger enhancement range between *t*_1_ and *t*_2_ make it possible to enhance the color contrast, setting the ranges too wide may cause over-enhancement. First, we analyzed the tone in *a∗* of images used in our animal experiment to determine [*s*_*n*_, *t*_*n*_] and found that the range of *a∗* is 15 < *a∗* < 50. Therefore, we tested [*s*_*0*_, *t*_*0*_] = [0, 0], [*s*_1_, *t*_1_], and [*s*_2_, *t*_2_] in a range between 15 and 50 and found that [*s*_1_, *t*_1_] = [15, 5] and [*s*_*2*_, *t*_*2*_] = [30, 30] show relatively good performance balancing the color contrast between red and white tone and naturalness which is the reproducibility of WLI image appearance.

Image examples are shown in Figures 2(a)–2(e), where Figures 2(a)–2(e) represent WLI, TXI mode2, TXI mode1, TXI mode2 without bright spot extraction from detail layer (6), and TXI mode1 without bright spot extraction from detail layer (6), respectively. As shown in Figure 2, when comparing TXI mode2 with WLI, the contrast of mucosal color and structure changes can be enhanced in TXI mode2, and the color appearance of TXI mode2 is close in characteristic to that of WLI. In addition, the brightness in dark areas is increased in TXI mode1 and mode2 while bright areas are preserved. Comparing TXI mode1 and mode2, mode1 has much higher mucosal color contrast especially between red and white color. The bright spots are enhanced in TXI without bright spot extraction from detail layer (6) in Figures 2(d) and 2(e) because of the enhancement of the detail layer including the bright spots. Conversely, the augmentation of such bright spots in TXI in Figures 2(b) and 2(c) can be suppressed by using equation (6).

### 2.2. Quantitative Assessment Metrics for Endoscopic Image Evaluation

Several quantitative assessment metrics are widely used to evaluate real-world image visibility. In endoscopic vision assessment, there are some studies in which the visibility has been evaluated by quantitative assessment [16, 22]. However, the subjective assessment by physicians is currently the primary way to validate image quality of gastrointestinal endoscopic images, and the establishment of the quantitative assessment is a challenging task since there are no available gold standards. In this work, we define the following quantitative assessment metrics for validating TXI performance of the texture, brightness, and color enhancement: (1) standard deviation of averaged illumination, (2) color difference, (3) edge-based contrast measure (EBCM) [23], and (4) structure similarity index (SSIM) [24].

We define standard deviation of averaged illumination as a metric of illumination uniformity. The metric can be interpreted as an indicator of brightness correction in dark image areas where the smaller the value is, the better the uniformity. Here, the averaged illumination of the image is derived using

(17) $$\begin{array}{c} \tilde{Y}\left(x,\;y\right)=F_{k}*Y\left(x,\;y\right), \end{array}$$

(18) $$\begin{array}{c} Y\left(x,\;y\right)=0.299I_{R}\left(x,\;y\right)+0.587I_{G}\left(x,\;y\right)+0.114I_{B}\left(x,\;y\right),\; \end{array}$$

where **Y** from RGB is derived by using parameters defined in the ITU-R BT.601 and **F**_*k*_ is averaging filter with kernel size *k* and *∗* is convolution operator. **F**_*k*_ is used for eliminating the effect of image noise and contrast on the metric of illumination uniformity. *k* is empirically determined. We tested *k* from 1 to 29, and the result in *k* = 17 is relatively consistent with the subjective result.

As mentioned above, the color difference Δ*E* has been used recently as the metric for the color contrast in gastrointestinal endoscopic images. Thus, in this work, we define the color difference as the metric for the color tone enhancement.

We define EBCM as an indicator for image contrast. EBCM is defined as the contrast between **I**(*x*, *y*) and its average edge-weighted value **E**(*x*, *y*) in a patch *O* which is a region of interest (ROI) for calculation of image contrast [16, 23]:

(19) $$\begin{array}{c} \text{EBCM}=G^{-1}\underset{\left(x,\;y\right)\in O}{\sum }\frac{\left|I\left(x,y\right)-E\left(x,y\right)\right|}{\left|I\left(x,y\right)+E\left(x,y\right)\right|}, \end{array}$$

(20) $$\begin{array}{c} E\left(x,y\right)=\frac{\sum_{\left(u,v\right)\in \Omega }g\left(u,v\right)I\left(u,v\right)}{\sum_{\left(u,v\right)\in \Omega }g\left(u,v\right)},\; \end{array}$$

where Ω is the set of all neighboring pixels of (*x*, *y*), *g* (*u*, *v*) is the edge value at pixel (*u*, *v*), and *G* is the total pixel number in ROI.

The SSIM is an evaluation metric proposed in [24]. SSIM is used for evaluating the similarity between the original image and enhanced image by evaluating image luminance, contrast, and structure. We use SSIM as the metric for naturalness, defined in our case as the reproducibility of WLI image appearance.

## 3. Experimental Results

### 3.1. Experimental Setting

The TXI algorithm was applied to endoscopic images obtained from animal testing. We acquired endoscopic images in the esophagus, stomach, and colon of anesthetized pigs for validating TXI performance. In this work, all images were obtained by using the EVIS LUCERA ELITE system and GIF-H290Z endoscope (Olympus Corporation, Tokyo, Japan). Raw images corresponding to the preprocessed image, i.e., image sensor output, were obtained. Reference images and enhanced images were generated from raw images by computer simulation ensuring identical scene and angle of incidence in the mucosa between methods. We defined the reference image as conventional WLI with structure enhancement level A3 and enhanced images as TXI mode1, TXI mode2, and conventional or clinically used enhancement methods such as structure enhancement level A8 and IHb color enhancement. Structure enhancement [9] is an endoscopic processor setting that increases the sharpness of coarse image features from low (1) to high (8). We set the level A3 as the reference image because that setting is the default setting of the EVIS LUCERA ELITE system. IHb color enhancement [9] is also a setting that increases color contrast based on a hemoglobin index in the image, and red color becomes more red and white color becomes whiter. In addition to these clinically used methods, we compared TXI with conventional techniques such as HE for real-world image processing and a newly proposed retinex-based technique M1 [16] for surgical endoscopic image augmentation. The structure enhancement setting of all enhanced images is A3 unless otherwise noted. All the experiments were conducted on a PC running Windows 10 professional 64-bit system utilizing Microsoft Visual Studio C++ 2012 and MATLAB 2019b. All animal experiments were performed with the approval of the animal ethics committee of Olympus Corporation, Tokyo, Japan.

### 3.2. Subjective Evaluations

The capability of TXI to selectively enhance brightness was assessed in images of the esophagus (Figure 3). The brightness in the center region is increased under TXI (Figures 3(d) and 3(g)) while the brighter peripheral area is maintained. Compared with reference (Figure 3(a)), HE (Figure 3(e)) and M1 (Figure 3(f)) are over-enhanced. In the HE image, while whole image contrast is increased but expansion of the dark region occurs. Brightness in the peripheral area is increased to an unnatural extent in M1 (Figure 3(f)). On the other hands, TXI (Figures 3(d) and 3(g)) can naturally enhance dark regions compared with HE and M1.

Next, the ability of TXI to enhance color contrast was assessed in endoscopic images of the stomach (Figure 4). The color contrast of TXI mode1 (Figure 4(g)) and mode2 (Figure 4(d)) appears higher than that of reference (Figure 4(a)) and IHb color enhancement (Figure 4(b)). In addition, white hues become whiter under TXI mode1, resulting in greater contrast between red and white tones particularly at the center of the image depicted as white dotted circles in Figure 4(g). HE and M1 [16] methods increase whole image contrast; however they also cause expansion of areas of halation (Figures 4(e) and 4(f), arrows).

Finally, texture enhancement by TXI in comparison with other methods was investigated. As shown in Figure 5, M1 (Figure 5(f)), TXI mode1 (Figure 5(g)), and mode2 (Figure 5(d)) have much better contrast, especially slight mucosal morphological changes, over reference (a), IHb color enhancement (b), HE (e), and A8 structure enhancement (c). While the M1 algorithm generates greater whole image contrast, it suffers from over-enhancement and halation is evident on the left side of the image (Figure 5(f)). On the other hand, TXI can naturally enhance slight mucosal contrast compared with M1 (Figures 5(d) and 5(g)).

### 3.3. Quantitative Evaluations

A quantitative evaluation of brightness, color, and texture enhancement was performed using three images as shown in Figure 6. All metrics except for color difference were calculated in the ROI depicted as a white square in each image. We set several ROIs as shown in Figure 7, for calculating the color difference ∆E between red and white color. ROIs depicted as red squares and white squares indicate the regions with red and white colors in each endoscopic image, respectively. The size of each ROI was set to 20 × 20 pixels. ∆E between averaged CIE 1976 La*∗*b*∗* values in each red and white ROI was calculated.

Table 1 shows the result of the quantitative evaluation of the seven image processing methods on different anatomic regions. The standard deviation of averaged illumination is used as a metric of illumination uniformity. As shown in Table 1, TXI mode1 has smaller values than the reference, IHb color enhancement, and the A8 structure enhancement images, and the two modes of TXI have almost the same value. Compared with HE and M1 [16], TXI has a smaller standard deviation of averaged illumination intensity. These results show that TXI mode1 and mode2 can reduce the nonuniformity of the image, by enhancing the brightness selectively in dark areas. Color difference ∆E is defined as a metric of color contrast. As shown in Table 1, TXI mode1 has higher ∆E than nearly all other enhancement methods. These results show that TXI can improve the visibility of color contrast between red and white colors over other enhancement methods. In addition, when comparing TXI mode1 with mode2, ∆*E* of mode1 is higher than that of the mode2, consistent with the algorithm design in which TXI mode1 adjusts color contrast while mode2 does not. The M1 image has greater color difference than TXI in the esophagus; however, as shown in Figure 3, M1 images tend to be overenhanced compared with other enhancement methods. In order to assess image contrast, EBCM resulting from each enhancement method is measured (Table 1). TXI mode1 and mode 2 have higher values than all other enhancement approaches showing that TXI can greatly enhance image contrast arising from texture enhancement. We finally show the result of the effect of TXI on naturalness of images. Higher values of SSIM in Table 1 indicate better naturalness preservation. IHb color enhancement has the highest SSIM value, indicating IHb color enhancement is most close to the reference. The SSIM value of TXI is relatively close to IHb color enhancement and A8 structure enhancement and much higher than HE and M1. TXI mode2 has higher SSIM value than TXI mode1 as predicted given its lack of color tone enhancement. These results are consistent with the subjective result (Figures 3–5), showing that TXI maintains much better naturalness over HE and M1, and TXI mode2 has better naturalness over TXI mode1.

## 4. Discussion and Summary

This paper presented an investigation to explore the possibility of implementing retinex-based enhancement in the chain of endoscopic image processing for potentially improving lesion visibility. Several studies in which retinex theory were utilized for enhancing endoscopic visibility have been reported [14–16], and the aim of these studies was primarily to enhance poor visibility due to physically limited (nonuniform and highly directional) illumination in endoscope. Conversely, the aim of this work is to improve not only the illumination nonuniformity in the image but also enhance subtle tissue differences by applying retinex-based algorithms to gastrointestinal images. The findings from the investigation are summarized as follows:

1. TXI can enhance brightness selectively in dark areas of endoscopic images and can enhance subtle tissue differences such as slight morphological and/or color changes over conventional enhancement methods including structure enhancement and IHb color enhancement.
2. Comparing TXI with a conventional technique (HE) for real-world image processing and newly proposed retinex-based technique for surgical endoscopic image augmentation [16], TXI can achieve significant image enhancement with characteristics of WLI appearance while preventing over-enhancement observed in these other methods.
3. TXI has two modes, mode1 and mode2, and enhancement of brightness and texture is similar between them. The enhancement of color contrast of the mode1 is superior to that of mode2 in accordance with the color enhancement of the mode1 algorithm; however, the naturalness in mode2 is better than that of the mode1.

Overall, TXI provides a balance of improving image features important for the physician searching for abnormalities (selective increase in brightness, greater color separation, and texture enhancement) while minimizing gross changes that may negatively impact familiarity (naturalness).

Although our proposed TXI algorithm outperforms other enhancement technologies, there are two main limitations. Firstly, SSR [17] was adopted in this work since it is a simple algorithm and easy to implement. However, the performance of SSR depends on the variance of the filter used for calculating the base layer, and we determined empirically that value for animal endoscopic images. Further investigation to check whether the performance of TXI can be improved by using an advanced retinex model reported in real-world image processing [25] is needed. The second limitation of this work is that only limited numbers of endoscopy cases in animals were conducted to validate the performance of the TXI algorithm, and the parameters of TXI were adjusted specifically for animal endoscopic images. Thus, the parameters are needed to be optimized for applying TXI to actual clinical endoscopic images obtained from humans. In addition, the consistency between the subjective evaluation and the proposed quantitative evaluation metrics was demonstrated only by the result obtained from these animal experiments. Therefore, further work is needed to check for agreement between the subjective evaluation from physicians and our proposed metrics described here.

We have described two TXI modes in this work. Our animal testing shows that the color contrast of TXI mode1 is much better than that of TXI mode2 since TXI mode1 directly expands color tone in La*∗*b*∗* space; however, the naturalness of TXI mode2 is better than that of TXI mode1. In actual clinical practice, maintaining color appearance close to WLI could be preferable to many physicians since current standard practice entails the use of WLI during inspection. Thus, it will be interesting to compare the performance of TXI mode1 and mode2 in actual clinical use.

We are now investigating the clinical relevance of the TXI algorithm by applying it to actual clinical endoscopic images obtained from upper and lower endoscopy. The results of this evaluation will be published in the near future. TXI can also be combined with optical image enhancement technology such as NBI since TXI is implemented entirely in the chain of endoscopic image processing. We are also now investigating the possibility of that combination for clinical practice. Moreover, deep learning-based methods are increasingly being applied to endoscopic images, particularly for improving lesion detection. Combination of such technologies and TXI is expected to improve detection performance since TXI can enhance subtle contrast over conventional WLI. In this regard, we have also explored the possibility of combining artificial intelligence and TXI and a report of this investigation is forthcoming.

## Figures and Tables

**Figure 1:** Flowchart of TXI.

**Figure 2:** Image examples. (a) WLI, (b) TXI mode2, (c) TXI mode1, (d) TXI mode2 without bright spot extraction from detail layer (6), and (e) TXI mode1 without bright spot extraction from detail layer (6).

**Figure 3:** Comparison of image processing methods for selective brightness enhancement in endoscopic images of the esophagus. (a) Reference (WLI with A3 structure enhancement), (b) IHb color enhancement, (c) A8 structure enhancement, (d) TXI mode2, (e) HE, (f) M1 [16], and (g) TXI mode1.

**Figure 4:** Comparison of image processing methods for color enhancement in endoscopic images of the stomach. (a) Reference (WLI with A3 structure enhancement), (b) IHb color enhancement, (c) A8 structure enhancement, (d) TXI mode2, (e) HE, (f) M1 [16], and (g) TXI mode1.

**Figure 5:** Comparison of image processing methods for texture enhancement in endoscopic images of the colon. (a) Reference (WLI with A3 structure enhancement), (b) IHb color enhancement, (c) A8 structure enhancement, (d) TXI mode2, (e) HE, (f) M1 [16], and (g) TXI mode1.

**Figure 6:** Quantitative evaluation images: (a) esophagus, (b) stomach, and (c) colon.

**Figure 7:** Assignment of ROIs for color difference calculation ∆E in images of (a) esophagus, (b) stomach, and (c) colon. Red and white squares represent ROIs for red and white color measurement, respectively.

**Table 1:** Quantitative evaluation of enhancement methods for image criteria improvement. Bold numbers represent the best or equally best performance in each metric.

Metrics	Scene	Reference (WLI w/A3)	IHb color enhancement [9]	WLI w/A8 [9]	HE	M1 [16]	Proposed TXI mode1	Proposed TXI mode2
Illumination uniformity (standard deviation)	Esophagus	37.165	39.134	37.323	60.222	58.102	**33.353**	33.643
	Stomach	**19.016**	20.979	**19.086**	33.759	26.553	19.108	19.293
	Colon	**19.315**	19.737	19.583	33.439	44.775	**19.344**	19.424
	Average	25.165	26.617	25.330	42.473	43.143	**23.935**	24.120

Color (ΔE)	Esophagus	8.004	9.120	9.586	15.221	**19.228**	16.026	13.474
	Stomach	4.471	5.055	5.102	7.619	7.441	**12.364**	8.542
	Colon	5.590	6.596	6.254	5.666	13.375	**15.407**	9.887
	Average	6.022	6.924	6.981	9.502	13.348	**14.599**	10.634

Contrast (EBCM)	Esophagus	5.264	5.244	9.117	8.898	6.319	**10.176**	**10.132**
	Stomach	5.167	5.175	8.839	7.780	6.630	**9.865**	**9.830**
	Colon	4.909	4.842	9.094	8.582	9.709	**9.829**	**9.856**
	Average	5.114	5.087	9.017	8.420	7.552	**9.957**	**9.939**

Naturalness (SSIM)	Esophagus	1.000	**0.995**	**0.970**	0.839	0.534	0.852	**0.926**
	Stomach	1.000	**0.996**	**0.977**	0.827	0.563	**0.916**	**0.957**
	Colon	1.000	**0.997**	**0.982**	0.836	0.029	**0.930**	**0.973**
	Average	1.000	**0.996**	**0.977**	0.834	0.375	0.899	**0.952**

## Data Availability

The data used to support the findings of this study are currently under embargo while the research findings are commercialized. The data can be available after the whole research is commercialized, and requests for data will be considered by the corresponding author.
